The article "Psychometric Assessment of the Persian Translation of the Interpersonal Mindfulness Scale With Undergraduate Students" was retracted in 2023. Reasons: signs of a paper mill; concerns about the authorship.

# Psychometric Assessment of the Persian Translation of the Interpersonal Mindfulness Scale With Undergraduate Students

**DOI:** 10.3389/fpsyt.2022.866816

**Published:** 2022-04-12

**Authors:** Abbas Abdollahi, Balachandran Vadivel, Dinh Tran Ngoc Huy, Maria Jade Catalan Opulencia, Pham Van Tuan, Abbas Abd Ali Abbood, Zarina Nasirova, Supat Chupradit, Kelly A. Allen, Olga Bykanova

**Affiliations:** ^1^Department of Counseling, Faculty of Education and Psychology, Alzahra University, Tehran, Iran; ^2^Department of English, Cihan University, Duhok, Iraq; ^3^Banking University HCMC, Ho Chi Minh City, Vietnam; ^4^International University of Japan, Niigata, Japan; ^5^College of Business Administration, Ajman University, Ajman, United Arab Emirates; ^6^National Economics University, Hanoi, Vietnam; ^7^Al Mustaqbal University College, Education Teaching Methods, Hillah, Iraq; ^8^Department of Internal Diseases, Samarkand State Medical Institute, Samarkand, Uzbekistan; ^9^Department of Occupational Therapy, Faculty of Associated Medical Sciences, Chiang Mai University, Chiang Mai, Thailand; ^10^Educational Psychology and Inclusive Education, Faculty of Education, Monash University, Clayton, VIC, Australia; ^11^Department of Higher Mathematics, Plekhanov Russian University of Economics, Moscow, Russia

**Keywords:** interpersonal mindfulness scale, undergraduate students, psychometrics, reliability, higher education, positive psychology

## Abstract

Interpersonal mindfulness is a construct that significantly contributes to social interaction. To date, no validated measure assessing interpersonal mindfulness has been developed in Iran. Therefore, the aim of this study was to translate and validate the Interpersonal Mindfulness Scale (IMS) among Iranian undergraduate students. Participants in the study (370 undergraduate students; 220 females) from the Azad University completed the translated IMS, the Five Facet Mindfulness Questionnaire, and the Inventory of Interpersonal Problems Scale. The translated measure demonstrated acceptable face validity. All items had acceptable content validity and were deemed essential to the scale. The results of a Confirmatory Factor Analysis (CFA) confirmed a scale with four subscales (presence, awareness of self and others, non-judgmental acceptance, and non-reactivity), with acceptable internal consistency. The findings support the psychometric properties of the Persian translated Interpersonal Mindfulness Scale, which could be used to measure interpersonal mindfulness among undergraduate students in Iran.

## Introduction

Young adulthood is considered a crucial phase in the course of human development often characterized by transition and change in social roles concerned with peers, employment, family, or further study (1, 2). Such changes have been found to be a stressor in young adulthood and attributed to the increase of mental health problems in this age group (3). The average-age onset of psychological problems such as depression, anxiety, as well as suicide ideation occur before the age of 24 years (4). Given the social-based changes that occurs in young adulthood due to life transitions and the importance of social support in this age group, interpersonal skills become important for relationship building and help seeking (4). Skills such as interpersonal mindfulness have been found to be an essential aspect of interpersonal competencies, yet remain largely unstudied. The purpose of this paper is to test the psychometric properties of the Persian translation of the interpersonal mindfulness scale.

The World Health Organization (WHO) defines mental health as having a positive attitude to achieve goals, being able to adapt to the social environment, having physical health, experiencing a sense of happiness and mental wellbeing, having effective interpersonal relationships with others, and coping effectively with problems (5). Mindfulness has been shown to positively influence the quality of relationships one may have across their personal, social, and work lives (6). Mindfulness is defined as the intentional attention of the present moment, observation as opposed to judgment, and acceptance of thoughts and feelings (7). Increasing research shows that mindfulness has positive effects on the individual, including increased meaning and satisfaction with their personal life, high self-efficacy, and the experience of positive emotions (8–10). Research shows a positive relationship between mindfulness and interpersonal skills such as empathetic communication (11), active listening (12), and establishing effective relationships with others (13).

However, in the field of positive psychology, there are very few reliable measures that cater for the interpersonal elements mindfulness (14). To address this gap, Pratscher et al. (15) developed the Interpersonal Mindfulness Scale (IMS), which measures the impact of mindfulness in interpersonal relationships. This 27-item scale uses four subscales to measure mindfulness: Presence (the ability to focus on interpersonal interactions with complete presence and accuracy), Awareness of Self and Others (the ability to pay attention to one's own inner experiences and those of others, including non-verbal behavior and intent), Non-judgmental Acceptance (the ability to accept and not prejudge interpersonal interactions), and Non reactivity (the ability to interact intelligently and avoid quick reactions). The English version of the IMS was first validated among 585 students in the United States (15). The results of an exploratory factor analysis found strong correlations between factors and support for the theoretical model. The validation of the 27-item IMS also showed strong reliability with a Cronbach's Alpha of 0.76 (16). Interpersonal mindfulness is a construct that is not related to the particular culture or region. Interpersonal mindfulness helps individuals to have effective interpersonal relationships and healthy and peaceful communications with others. Therefore, this measure was chosen to do the psychometric study among Iranian population.

Various validated measures have been designed to assess mindfulness, including the Freiburg Mindfulness Inventory (17), the Toronto Mindfulness Scale- trait version (18), and the Mindful Attention Awareness Scale (19). These measures are designed to assess the construct of mindfulness more broadly and do not measure the impact of mindfulness in interpersonal relationships. The IMS is the first psychometric tool to measure interpersonal mindfulness (16). Therefore, mindfulness scales focus on the individual, and the IMS seeks to use the benefits of mindfulness in interpersonal relationships. Individuals with high levels of interpersonal mindfulness maintain their awareness during interpersonal interactions and are aware of their emotions, feelings, thoughts and experiences during the interactions with others. They also pay attention to the other person's feelings, thoughts, verbal tone and body language. They are good listeners and talkers during interaction with others (15).

Considering the pivotal role that interpersonal skills play in mental health, relationship building and transition to adulthood, as well as the importance of interpersonal mindfulness for relationship skills and satisfaction, the use of appropriate measures that evaluate interpersonal mindfulness are important for future research, education, and preventative interventions in the field of positive psychology and higher education. There is currently no measure in Iran that assesses interpersonal mindfulness. Therefore, the present study aimed to translate the IMS into Persian and validate the scale in order to enhance the quality of interpersonal interactions, contribute to the research literature, and to assist Iranian researchers and psychotherapists in measuring interpersonal mindfulness. The purpose of this research was therefore to examine the psychometric properties of the Persian version of the Interpersonal Mindfulness Scale in a sample of Iranian youth.

## Methods

### Participants

Participants in this study were 370 undergraduate students (220 females and 150 males) from Azad University, Tehran, Iran. The participants ranged in age from 18 to 24 years (*M* = 20.12, *SD* = 3.86). The majority of participants were single (*N* = 275), and the rest were married (*N* = 95). One-hundred and nineteen (30%) participants were from medical fields, 107 (29%) participants were from technical fields, and 144 (39%) participants were from social science fields. In terms of academic year, 129 (35%) students were in the first year of university, 118 (32%) students were in their second year, 74 (20%) students were in their third year, and 49 (13%) students were in the last year of university. Inclusion criteria in this study included undergraduate students, those between the age of 18 and 24.

### Instruments

#### Interpersonal Mindfulness Scale [IMS]

The IMS consists of 27 items and evaluates four subscales: Presence (e.g., *Rather than being distracted, it is easy for me to be in the present moment while I am interacting with another person*), Awareness of Self and Others (e.g., *When I am with other people, I am aware of my moods and emotions*), Non-judgmental Acceptance (e.g., *When in a discussion, I accept others have opinions different from mine*), and Non-reactivity (e.g., *When I receive an angry text/email from someone, I try to understand their situation before responding*). This measure is based on a 5-point Likert scale from 1 (*almost never*) to 5 (*almost always*), with a greater score in each subscale indicating a higher level of the subscale (e.g., greater presence). One previous study reported an acceptable internal consistency with a Cronbach's Alpha of 0.76 (16).

Initially, the permission was obtained from the developer of the IMS. The Brislin (20) translation method was employed in order to translate the English version of the IMS into Persian. Two experienced translators who were fluent in English and Persian were independently invited. The translation of the IMS measure from English into Persian was first conducted by one translator. The second translator was then asked to back-translate the resulting measure from Persian into English, unaware of the first translation operation. Finally, the two versions were compared by three independent translators and no major variations in terms of content and concept between the Persian version measure and the original version measure were found.

#### Five Facet Mindfulness Questionnaire [FFMQ]

This measure assesses individual mindfulness with 39 items across five subscales: non-reactivity to inner experiences (e.g., *I perceive my feelings and emotions without having to react to them*), observing or attending to sensations (e.g., *I notice how my emotions express themselves through my body*), acting with awareness (e.g., *I find myself preoccupied with the future or the past; reverse scored*), describing (e.g., *I'm good at finding the words to describe my feelings*), and non-judging of experience (e.g., *I disapprove of myself when I have irrational ideas; reverse scored*) (21). This measure uses a 5-point Likert scale from 1 (never or very rarely true) to 5 (very often or always true), with a greater score indicating a greater level of mindfulness. In this study, an Persian version of this measure was used which had previously been found to have an acceptable internal consistency with a Cronbach's Alpha of 0.83 (22).

#### Inventory of Interpersonal Problems Scale [IIPS]

The IIPS measures difficulty in interpersonal relationships using 32 items across eight subscales: domineering (e.g., *It is hard for me to understand another person's point of view*), vindictive (e.g., *It is hard for me to be supportive of another person's goals in life*), cold (e.g., *It is hard for me to show affection to people)*, socially avoidant *(e.g., It is hard for me to join in groups)*, nonassertive *(e.g., It is hard for me to tell a person to stop bothering me)*, exploitable *(e.g., It is hard for me to let other people know when I am angry)*, overly nurturant *(e.g., It is hard for me to attend to my own welfare when somebody else is needy)*, and intrusive *(e.g., It is hard for me to keep things private from other people)* (23). This measure is based on a 5-point Likert scale from 0 (*not at all*) to 4 (*extremely*), and a greater score indicates a greater level of difficulties in interpersonal relationships. In this study, an Persian version of this measure was used and reported an acceptable internal consistency with Alpha Cronbach of 0.83 (24).

### Ethical Considerations

The study process was reviewed and approved by the ethics committee of Alzahra University, Tehran, Iran. After reviewing the research objectives and questionnaires, Azad University permitted to distribute the questionnaires among undergraduate students. Written consent forms were signed by participants prior to completing the questionnaires.

### Procedure

Participants were recruited via a multistage cluster random sampling method. In the first step, thirteen faculty members were identified from three disciplines, including social sciences, technical, and medicine. One faculty member from each discipline was randomly selected, and one class from each selected faculty member was randomly chosen. Questionnaires were distributed among the students of that class. The data collection occurred throughout the month of December 2019. Questionnaires took participants about 45 min to complete, with a 5-min break with a refreshment (including cake and drinks) occurring mid-way through. Inclusion criteria for participation in this study including being a bachelor's (undergraduate) student, being in the age range of 18–24 years, and being willing to participate in the study. Fifteen questionnaires were removed from the dataset due as these participants were over 24 years old.

### Data Analyses

Face validity technique was employed to explore comprehensibility and relevance of items to the construct based on subjective judgment. The impact score [frequency (%) × importance] was employed to determine relevancy, comprehensibility, and the appropriateness of items to the construct using a 5-point Likert scale rated from 1 (*not important*) to 5 (*completely important*). Frequency refers to the number of participants who chose options 4 and 5 on the scale. Importance refers to the average score of each item. If the value of the impact score is greater than the cut-off score of 1.5, it can be concluded that the item has acceptable face validity (25).

Content validity technique was employed to consider the appropriateness of items to the specific construct. The Content Validity Index (CVI) was employed to measure simplicity, clarity, and relevance via a 4-point Likert scale from (1) *not relevant at all* to (4) *highly relevant*. The value of the CVI is calculated by dividing the number of experts who selected “3” and “4” by the total number of experts. The item has acceptable content validity if the CVI value is equal to or >0.7 (26). The Content Validity Ratio (CVR) was employed to measure the essentiality of items via a 3-point Likert scale from (1) *not essential* to (3) *essential* (26). The value of CVR is calculated as follows: The number of experts who select the value of “3” minus half the number of experts is divided by half the number of experts. A CVR value greater than Lawshe's value (.62) indicates satisfactory content validity for the item (27).

To estimate construct validity, a confirmatory factor analysis in AMOS software was used to analyze the hypothesized relationships between the items and the factors. Regarding sample size for the confirmatory factor analysis, Hair et al. (28) recommended a ratio of cases to items of 10:1. In this study, there were 370 cases as well as 27 items, and the minimum ratio of cases to items is met. Construct validity is evaluated in three steps:

(a) Evaluation of factor loadings: Factor loading values must be >0.5, <1, and non-negative (29).
(b) Evaluation of the measurement model fit indices: CMIN/df < 5; Root Mean Squared Error of Approximation (RMSEA) < 0.08; Tucker- Lewis Index (TLI), Comparative Fit Index (CFI), and the Goodness of Fit Index (GFI) > 0.90 (30).
(c) Evaluation of convergent validity and internal consistency: Average Variance Extracted (AVE) was used to measure convergent validity. An AVE value > 0.5 indicates the items of the construct do not violate convergent validity cutoffs. Construct Reliability (CR) and omega were used to measure the internal consistency of the measure. The construct has acceptable internal consistency if the values of CR and omega ate > 0.7 (30, 31).

### Preliminary Analysis

Statistical Package for the Social Science (SPSS version 24) and Asset Management Operating System (AMOS version 24) were employed to analyze the data. Preliminary analyses, such as missing data, outliers, and normality, were evaluated using SPSS, and a confirmatory factor analysis was conducted using AMOS.

## Results

### Face Validity

To evaluate the face validity of each item, 15 participants evaluated the relevancy, comprehensibility, and appropriateness of items on a 5-point Likert scale. The impact score was calculated, and the results showed that the impact scores for all items were above 1.5, indicating the items had acceptable face validity.

### Content Validity

Ten experts (psychologists) were recruited to estimate the content validity of each item. As seen in Table 1, the values of CVI were above the acceptable cut-off score of 0.7, indicating all items had acceptable content validity. As see in Table 1, the values of CVR were greater than the cut-off score given by Lawshe's table (0.62), indicating each item was essential (27).

**Table 1:** CVR and CVI for the items of Interpersonal mindfulness scale.

**No**	**Items**	**CVI**			**CVR**
		**Simplicity (1–4)**	**Relevancy (1–4)**	**Clarity (1–4)**	**Essential (1–3)**
1	When I am with other people, I am aware of my moods and emotions.	0.89	1	1	0.93
2	When I am conversing with another person, I am fully engaged in the conversation.	0.92	1	0.98	1
3	When in a discussion, I accept others have opinions different from mine.	0.96	1	1	0.85
4	In tense moments with another person, I am aware of my feelings but do not get taken over by them.	1	1	1	1
5	When a person is talking to me, I find myself thinking about other things, rather than giving them my full attention.	1	1	1	1
6	When I receive an angry text/email from someone, I try to understand their situation before responding.	1	1	1	0.83
7	I listen for the meaning behind another person's words through their gestures and facial expressions.	0.91	0.89	1	1
8	When I am upset with someone, I notice how I am feeling before responding.	1	0.89	0.87	0.99
9	I listen carefully to another person, even when I disagree with them.	0.94	1	0.86	0.97
10	I find myself listening to someone with one ear while doing something else at the same time.	1	1	1	1
11	I take time to form my thoughts before speaking.	1	1	1	1
12	I think about the impact my words may have on another person before I speak.	1	1	1	1
13	When interacting with someone I know, I am often on autopilot, not really paying attention to what is actually happening in the moment.	0.97	1	0.93	1
14	When I am with another person, I try to accept how they are behaving without wanting them to behave differently.	1	1	1	1
15	I am aware of others moods and tone of voice while I am listening to them.	1	1	1	1
16	I am aware of my facial and body expressions when interacting with others.	1	1	1	0.86
17	When I am with others, I am easily distracted and my mind tends to wander.	1	1	1	1
18	When interacting with others, I am aware of their facial and body expressions	1	1	1	1
19	I pick up on the intentions behind what another person is trying to say.	0.88	0.94	1	1
20	I listen to another person without judging or criticizing them.	0.89	1	0.87	1
21	I give the appearance of listening to another person when I am not really listening.	0.93	0.94	1	1
22	Before I speak, I am aware of the intentions behind what I am trying to say.	1	0.99	1	1
23	When I am interacting with another person, I get a sense of how they are feeling.	1	1	1	0.86
24	I accept that another person's current situation or mood might influence their behavior.	1	1	1	1
25	Rather than being distracted, it is easy for me to be in the present moment while I am interacting with another person.	1	1	1	1
26	When speaking to another person, I am aware of how I feel inside.	1	1	1	1
27	I notice how my mood affects how I act toward others.	1	0.98	1	0.88

*CVR for an item was evaluated using the formula: $CVR=\frac{ne-N/2}{N/2}$. The N here denotes the number of experts and ne is the number of experts that scored 3 for the particular item*.

*The following formula was used for calculating the CVI: $CVI=\frac{ne}{N}$. Here, ne denotes the number of experts who scored 3 or higher for the particular item and N is the total number of participants/experts*.

### Construct Validity

The results of the preliminary analyses showed that the ratio of missing data to the total data was 2%, which was addressed using the regression imputation method. A box plot was used to evaluate univariate outliers and 10 questionnaires were excluded. The normality of the data was examined by the skewness and kurtosis, which have acceptable cutoff values of ±2 and ±3, respectively (32). Skewness values ranged between −1.21 and 1.11 and kurtosis values ranged between 1.23 and 2.34, indicating that the data was normally distributed.

Construct validity examines the empirical evidence in support of the hypothesized relationships between the items and the dimensions of the construct validity is evaluated in three steps:

(a) Evaluation of factor loadings: As seen in Figure 1, the factor loading values did not violate these criteria, therefore all items remained in the questionnaire. Table 2 shows the mean and standard deviation of each item.
(b) Evaluation of the measurement model fit indices: The results showed that the fit indices met the cut-off scores (CMIN/df = 3.71, *p* < 0.01, CFI = 0.91, RMSEA = 0.07, TLI = 0.90, GFI = 0.90), and confirmed the four subscales of the translated IMS.
(c) Evaluation of convergent validity and internal consistency: As seen in Table 3, the values of AVE, omega and CR are above the cut-off scores of 0.5 and 0.7, respectively, indicating satisfactory convergent validity and internal consistency for the translated IMS.

**Figure 1:** Confirmatory factor analysis with factor loadings for the four sub scales of IMS scale (*p* < 0.01).

**Table 2:** Means and standard deviations of the items of MIS.

**No**	**Items**	**Mean**	**Std. deviation**
1	When I am with other people, I am aware of my moods and emotions.	4.09	0.97
2	When I am conversing with another person, I am fully engaged in the conversation.	3.88	0.95
3	When in a discussion, I accept others have opinions different from mine.	2.29	1.10
4	In tense moments with another person, I am aware of my feelings but do not get taken over by them.	3.56	1.08
5	When a person is talking to me, I find myself thinking about other things, rather than giving them my full attention.	3.49	1.34
6	When I receive an angry text/email from someone, I try to understand their situation before responding.	4.25	0.84
7	I listen for the meaning behind another person's words through their gestures and facial expressions.	3.75	1.20
8	When I am upset with someone, I notice how I am feeling before responding.	3.96	1.18
9	I listen carefully to another person, even when I disagree with them.	3.89	1.23
10	I find myself listening to someone with one ear while doing something else at the same time.	3.71	1.26
11	I take time to form my thoughts before speaking.	3.39	1.15
12	I think about the impact my words may have on another person before I speak.	3.54	1.04
13	When interacting with someone I know, I am often on autopilot, not really paying attention to what is actually happening in the moment.	3.24	1.17
14	When I am with another person, I try to accept how they are behaving without wanting them to behave differently.	3.46	1.02
15	I am aware of others moods and tone of voice while I am listening to them.	3.57	1.32
16	I am aware of my facial and body expressions when interacting with others.	3.99	1.16
17	When I am with others, I am easily distracted and my mind tends to wander.	3.79	1.28
18	When interacting with others, I am aware of their facial and body expressions	2.92	1.05
19	I pick up on the intentions behind what another person is trying to say.	3.40	1.13
20	I listen to another person without judging or criticizing them.	3.41	1.17
21	I give the appearance of listening to another person when I am not really listening.	4.05	1.14
22	Before I speak, I am aware of the intentions behind what I am trying to say.	3.88	1.17
23	When I am interacting with another person, I get a sense of how they are feeling.	3.99	1.15
24	I accept that another person's current situation or mood might influence their behavior.	3.87	1.23
25	Rather than being distracted, it is easy for me to be in the present moment while I am interacting with another person.	3.77	1.13
26	When speaking to another person, I am aware of how I feel inside.	4.04	1.11
27	I notice how my mood affects how I act toward others.	3.44	1.23

Presence items: 2, 5*, 10*, 13*, 17*, 21*, 25. Awareness of self and others items: 1, 7, 15, 16, 18, 19, 23, 24, 26, 27. Non-judgmental Acceptance items: 3, 9, 14, 20. Non-reactivity items: 4, 6, 8, 11, 12, 22.

**Table 3:** AVE and CR for four subscales of IMS.

**Variable**	**AVE**	**CR**	**Omega**
Presence	0.50	0.72	0.74
Awareness of Self and Others	0.64	0.76	0.79
Non-judgmental Acceptance	0.64	0.78	0.81
Non-reactivity	0.94	0.87	0.90
Interpersonal mindfulness scale	0.68	0.85	0.88

### Convergent Validity

A correlation analysis was used to measure the convergent validity of the translated IMS with other measures. The results showed that the four subscales of IMS had negative relationships with the Inventory of Interpersonal Problems Scale and positive relationships with the Five Facet Mindfulness Questionnaire (see Table 4).

**Table 4:** Correlations between the studied variables.

**Variables**	**1**	**2**	**3**	**4**	**5**	**6**	**7**
1) Presence	1						
2) Awareness of self and others	0.82	1					
3) Non-judgmental acceptance	0.82	0.78	1				
4) Non-reactivity	0.78	0.81	0.84	1			
5) interpersonal problems	−0.71	−0.68	−0.66	−0.62	1		
6) five facet mindfulness	0.67	0.63	0.61	0.69	−0.56	1	
7) Interpersonal mindfulness	0.8	0.99	0.64	0.31	−0.64	0.63	1

*Correlation is significant at the 0.01 level*.

### Moderation Test of Fields of Study

In order to compare between three different fields of study (medical, technical and social science) in the proposed model, multi-group analysis was performed. The findings revealed that the fit indices for the variant-group model (χ^2^ = 6.21, *p* < 0.01, *RMSEA* = 0.19, *CFI* = 0.69, *GFI* = 0.74, *NFI* = 0.75) did not better than the fit indices of the invariant-group model (χ^2^ = 5.19, *p* < 0.01, *RMSEA* = 0.21, *CFI* = 0.73, *GFI* = 0.78, *NFI* = 0.79), suggesting that fields of study did not moderate the proposed model.

## Discussion

This study aimed to evaluate the validity and reliability of the Persian version of the Interpersonal Mindfulness Scale (15) in a sample of Iranian youth. The results demonstrated that the translated measure had acceptable psychometrics, including face, content, construct, and concurrent validity. The findings also showed that interpersonal mindfulness could be assessed using the IMS based on individuals' self-reports.

The IMS translation was performed using the Brislin method and the translators agreed on the consistency of the Persian edition of the IMS with the original version. The results of the content validity analysis showed that the experts agreed the 27 items of the IMS had acceptable content validity, which is consistent with the original study by Pratscher et al. (15). The face validity results showed that the items of the translated IMS had sufficient appropriateness, clarity, and comprehensibility. The results of the construct validity confirmed the measurement fit indices for the IMS and all items had acceptable factor loadings ranging from .44 to .99. The present study confirmed the four-factor structure of the measure, including presence, awareness of self and others, non-judgmental acceptance, and non-reactivity (15, 16). The results of the construct reliability analysis showed the translated IMS had acceptable internal consistency, with values from 0.72 (presence) to 0.87 (non-reactivity), which is consistent with the original study (15).

The present study is the first study to examine the psychometric properties of the IMS in an Iranian context. Two questionnaires [FFMQ and IIPS; (21, 23)] were used to examine concurrent validity. The results indicated that the IMS had a significant negative correlation with the IIPS and a significant positive correlation with the FFMQ. Mindfulness in interpersonal relationships is an important factor for understanding and monitoring behavior. Individuals who are mindful in their interactions have the ability to communicate effectively with others because they are able to be present in the moment and ignore distractions (33, 34). The results also showed a positive correlation between the components of the IMS and the components of the FFMQ. Interpersonal mindfulness can be viewed as a sense of being engaged and present in the moment, including the awareness and acceptance of thoughts and emotions related to self and others within an interpersonal interaction (35).

## Limitations

It should be noted that there are limitations of the present study in addition to the strengths of the scale. One of the limitations of this study was the limited demographics of the participants of the study. Future research should examine the strength of this scale in measuring interpersonal mindfulness among other age groups and clinical samples. Further research is needed to determine if the translated IMS is useful for those suffering from interpersonal problems, including social phobias and other disorders and whether it can be used as a tool in other age groups given the potential utility of interpersonal mindfulness for relationship building and a sense of belonging across the life space. This study was performed on undergraduate students. Future studies could be conducted on individuals with more or less academic levels. Although the results of CFA were the same as the original study' results. It is better future studies conduct exploratory factor analysis, because the measure was translated into the Persian language and used in Iran.

## Conclusions

According to the findings of the present study, the IMS had acceptable psychometric qualities, which suggests it is a suitable scale for measuring interpersonal mindfulness in Iranian youth. Therefore, this short scale, with its ease of implementation and desirable psychometric properties, can be used to evaluate interpersonal mindfulness in order to establish desirable social connections and shape interpersonal behaviors. Findings suggests that the IMS may have utility for researchers and psychologists interested in interpersonal skills.

## Data Availability Statement

The datasets presented in this study can be found in online repositories. The names of the repository/repositories and accession number(s) can be found below: the data is available on the figshare repository website doi: 10.6084/m9.figshare.14068241.

## Ethics Statement

The studies involving human participants were reviewed and approved by Alzahra University 14001113A. The patients/participants provided their written informed consent to participate in this study.

## Author Contributions

All authors listed have made a substantial, direct, and intellectual contribution to the work and approved it for publication.

## Conflict of Interest

The authors declare that the research was conducted in the absence of any commercial or financial relationships that could be construed as a potential conflict of interest.

## Publisher's Note

All claims expressed in this article are solely those of the authors and do not necessarily represent those of their affiliated organizations, or those of the publisher, the editors and the reviewers. Any product that may be evaluated in this article, or claim that may be made by its manufacturer, is not guaranteed or endorsed by the publisher.
